# Effects of surgery and anesthetic choice on immunosuppression and cancer recurrence

**DOI:** 10.1186/s12967-018-1389-7

**Published:** 2018-01-18

**Authors:** Ryungsa Kim

**Affiliations:** Breast Surgery, Hiroshima Mark Clinic, 1-4-3F, 2-chome, Ohte-machi, Naka-ku, Hiroshima, Japan

**Keywords:** Cancer surgery, Anesthetic agent, Anesthetic technique, Immunosuppression, Cancer recurrence

## Abstract

**Background:**

The relationship between surgery and anesthetic-induced immunosuppression and cancer recurrence remains unresolved. Surgery and anesthesia stimulate the hypothalamic–pituitary–adrenal (HPA) axis and sympathetic nervous system (SNS) to cause immunosuppression through several tumor-derived soluble factors. The potential impact of surgery and anesthesia on cancer recurrence was reviewed to provide guidance for cancer surgical treatment.

**Methods:**

PubMed was searched up to December 31, 2016 using search terms such as, “anesthetic technique and cancer recurrence,” “regional anesthesia and cancer recurrence,” “local anesthesia and cancer recurrence,” “anesthetic technique and immunosuppression,” and “anesthetic technique and oncologic surgery.”

**Results:**

Surgery-induced stress responses and surgical manipulation enhance tumor metastasis via release of angiogenic factors and suppression of natural killer (NK) cells and cell-mediated immunity. Intravenous agents such as ketamine and thiopental suppress NK cell activity, whereas propofol does not. Ketamine induces T-lymphocyte apoptosis but midazolam does not affect cytotoxic T-lymphocytes. Volatile anesthetics suppress NK cell activity, induce T-lymphocyte apoptosis, and enhance angiogenesis through hypoxia inducible factor-1α (HIF-1α) activity. Opioids suppress NK cell activity and increase regulatory T cells.

**Conclusion:**

Local anesthetics such as lidocaine increase NK cell activity. Anesthetics such as propofol and locoregional anesthesia, which decrease surgery-induced neuroendocrine responses through HPA-axis and SNS suppression, may cause less immunosuppression and recurrence of certain types of cancer compared to volatile anesthetics and opioids.

## Introduction

Surgical resection is the most effective method to remove primary tumors and metastatic lymph nodes. However, some cancer cells may remain after surgery, and micro-metastases or tumor dislodged during surgical manipulation may spread via lymphovascular vessels [1]. During the perioperative period, surgery induced stress responses and anesthetic-induced immunosuppression may play a critical role in establishment and growth of metastatic lesions [2–5]. Because immune responses are regulated by the hypothalamic–pituitary–adrenal (HPA) axis and sympathetic nervous system (SNS), surgery-induced or anesthesia-induced activation of these two systems may facilitate metastasis through several tumor-derived soluble factors [6].

HPA-axis and SNS activation suppress cell-mediated immunity (CMI) and release of catecholamines and prostaglandin E_2_ (PGE_2_). These factors, in turn, increase immunosuppressive cytokines, soluble factors (e.g., interleukin 4 [IL-4], IL-10, transforming growth factor beta [TGF-β], and vascular endothelial growth factor [VEGF]), and proinflammatory cytokines (e.g., IL-6 and IL-8), which promote tumor angiogenesis and metastasis [7–11]. Furthermore, volatile anesthetics and opioids suppress CMI and promote cancer cell proliferation and angiogenesis, whereas propofol inhibits tumor angiogenesis and does not suppress CMI [12, 13]. Regional anesthesia (RA) preserves CMI and decreases surgery-induced neuroendocrine responses by attenuating afferent neural transmission activation of the HPA-axis and SNS response. Thus, reduction in opioid and volatile anesthetic use may reduce cancer recurrence [14].

Clinically, the key question of whether anesthetic choice affects cancer outcome remains unresolved. Retrospective studies and meta-analyses suggest that particular anesthetic techniques may reduce cancer related mortality and recurrence by decreasing immunosuppression after surgical treatment for certain types of cancer [15]. Several prospective randomized controlled trials (RCTs) to define the effect of anesthesia on cancer recurrence are currently underway [15]. The present study relied on preclinical study review to determine the potential effects of surgery and anesthetic choice on immunosuppression and cancer outcomes to help guide treatment choices by clinicians and cancer surgeons.

## Perioperative period and immune function

The perioperative period is divided into three phases: the preoperative period (a few preoperative hours), the intraoperative period, and the postoperative period (several days after surgery) (Fig. 1a). During the intraoperative period, general anesthesia consists of administration of intravenous anesthetics (e.g., thiopental or propofol) for induction, followed by muscle relaxants and endotracheal intubation, then volatile anesthetics (e.g., sevoflurane) and opioids for maintenance and pain control. In contrast, RA uses a local anesthetic (e.g., lidocaine or bupivacaine) to block peripheral or spinal nerve transmission to produce a paravertebral or epidural block. Local anesthetics prevent surgical pain and reduce surgery-induced neuroendocrine stress by suppressing afferent neural transmission to the central nervous system. Thus, HPA-axis and SNS responses are avoided. Anesthetic choices during cancer surgery positively or negatively affect immune function during the perioperative period, and this immune balance may play a key role in cancer spread and recurrence (Fig. 1b).

**Fig. 1:** Perioperative period and immune balance. **a** The perioperative period includes the preoperative period, intraoperative period, and postoperative period. During these periods, several anesthetics agents and techniques may affect immune response and cancer recurrence after surgery. **b** Immune balance during the perioperative period is achieved through control of positive effects from regional anesthesia, propofol, and local anesthetics, with negative effects from volatile anesthetics, thiopental, and opioids. The immune balance needs to be shifted toward positive effects to reduce immunosuppression, which promotes cancer metastasis

Tumors release soluble factors into their microenvironments to block CMI surveillance and facilitate tumor growth and metastasis [16]. Soluble factors affect residual cancer cells and pre-existing micro-metastases to promote new metastases, which are the major cause of cancer-related death if not eliminated by immune cells [17–19]. In these situations, the perioperative period is pivotal in determining cancer outcomes following primary surgical treatment. Surgery, anesthesia, analgesia, and specific agents all influence immune function and tumor metastasis [19]. Immunosuppression arises within a few hours of surgery and lasts for several days, in proportion to the extent of surgical trauma. Although the immune system normally protects against tumor development, surgery-induced stress counteracts the anti-metastatic effects of CMI to allow dissemination and metastasis of cancer cells during and following surgery [12]. The perioperative period may be crucial to residual cancer cell spread, with anesthetic-induced immunosuppression affecting cancer recurrence and long-term prognosis [13, 14].

## Effect of surgery on immune function and tumor metastasis

Although surgical resection is a major component of cancer treatment, surgery itself suppresses immunity; thus, metastasis is promoted through growth facilitation of pre-existing micro-metastases and dissemination of cancer cells during resection of the primary lesion [20]. Detection of tumor cells in peritoneal blood and fluid after surgery has been associated with significantly shorter disease-free survival in patients with colorectal cancer [1, 21]. Given that surgery modifies neural, endocrine, metabolic, inflammatory, and immunologic microenvironments [22], surgery-induced stress responses may activate angiogenesis and increase vascularization to promote tumor growth [2–5].

Additionally, surgical resection may promote tumor growth and metastasis through increased matrix metalloproteinase 9 (MMP-9) and VEGF expression, as in one model of breast cancer [23]. Plasma VEGF levels are increased by surgery-induced stress during laparotomy and mastectomy [2], whereas TGF-β plasma levels decrease in response to lung metastasis in animal models [24]. Acceleration of metastasis after surgical resection through proliferation of distant, dormant micro-metastases has been observed in patients with breast cancer [25].

Primary tumor resection may directly stimulate cancer cell spread through metastatic lesion growth. Following surgical resection of a primary tumor, decreased endostatin and angiostatin levels allow new blood vessel growth, which promotes growth or metastatic lesions and uncontrolled proliferation [26]. Following primary colorectal tumor resection, decreased angiostatin and endostatin levels in urine and plasma are associated with increased metabolic activity in liver metastases [27]. Thus, it seems that the primary tumor inhibits angiogenesis for distant metastases, but that primary tumor resection allows for neovascularization and increased metabolic activity in metastases [25]. If surgery-induced immunosuppression occurs, surgery may fail to prolong survival in patients with cancer. Surgery reduces levels of endogenous antiangiogenic factors such as endostatin and angiostatin while weakening the immune surveillance needed to inhibit the growth of metastatic lesions [28].

Changes to NK cell activity depend on both the degree of surgical treatment and the intensity of the surgical stress response [29], which activates the HPA-axis and SNS to release catecholamines and prostaglandins [30]. Laparotomy increases lung tumor retention (LTR), whereas combined β-adrenergic antagonism and cyclooxygenase (COX) inhibition decrease LTR and restore NK cell function in experimental animal models [31]. Clinically, surgery decreases circulating NK and T cells through the programmed death-1 (PD-1) and programmed death–ligand 1 (PD-L1) pathway, due to increased caspase-3 activity in association with PD-1 expression on immune cells [32]. Surgical stress increases Th2 cells and decreases Th1 cells, which decreases the Th1/Th2 ratio and eventually suppresses CMI [33]. During surgical stress, levels of immune stimulating cytokines such as IL-2, IL-12, and interferon-γ (IFN-γ) are decreased, whereas anti-inflammatory cytokines such as IL-10 are increased [33]. The magnitude of immunosuppression is in proportion to the extent of surgical treatment. The overall effect of surgery on immune function and tumor metastasis is summarized in Table 1.

**Table 1:** Effect of surgery on immune function and tumor metastasis

Factor	Experimental data	Clinical data
Surgery-induced stress	Increased vascularization [3] Augmentation of angiogenesis [2] Inadvertent dispersal of tumor cells [20]	Modification of neural, endocrine, metabolic, inflammatory, and immunologic microenvironments [1] Detectable tumor cells in blood and peritoneal fluid after surgery associated with shorter disease-free survival in colorectal cancer [1] Surgery causes neoplastic cells to be dislodged from primary tumor [1, 21] Induction of angiogenesis and proliferation of distant, dormant micro-metastases in breast cancer surgery [4] Surgery-induced angiogenesis in breast cancer [5] Acceleration of metastasis by surgical resection of primary breast cancer [25]
Surgical manipulation		
NK cell activity	Suppression of NK cell activity, dependent on extent of surgical trauma and intensity of stress response [29] Stimulation of the hypothalamic-pituitary-adrenal (HPA) axis and the sympathetic nervous system Release of catecholamines and prostaglandins [30] Laparotomy associated with a significant increase in LTR [31] Combination of beta-antagonism and COX inhibition reduces LTR and restores NK cell function [31]	Decrease in circulating NK cell levels [32] Decrease in dendritic cells, CTLs, and T-helper cells [32, 33] Decrease in the Th1/Th2 ratio [33] Increase in pro-inflammatory cytokines (e.g., IFN-α, IL-6) [32] Increased cortisol and catecholamines [32] Magnitude of immunosuppression is proportional to degree of surgical manipulation [33]
Cell-mediated immunity		
Cytokines		
Others		
MMPs	Promotion effect on tumor growth and pulmonary metastasis of human breast cells by surgical process [23] Increased plasma VEGF levels induced by surgical stress [2, 23] Decreased plasma levels in lung cancer metastasis [24] Reduction of growth control factors endostatin and angiostatin [28]	Decrease in circulating anti-angiogenic factors angiostatin and endostatin after surgical resection of primary colorectal carcinoma [27] Regional anesthesia combined with propofol attenuates effect of breast surgery on MMPs compared to balanced general anesthesia with opioid anesthesia [48] Surgery induces a transient endostatin decrease in colorectal carcinoma [26] Decrease in circulating anti-angiogenic factors angiostatin and endostatin after surgical resection of primary colorectal carcinoma coincides with increased metabolic activity of liver metastases [27]
VEGF		
TGF-β		
Endostatin and angiostatin		

*NK* natural killer; *CTL* cytotoxic T-lymphocyte; *IL* interleukin; *Th1* T-helper 1; *Th2* T-helper 2; *IFN* interferon; *LTR* lung tumor retention; *COX* cyclooxygenase; *VEGF* vascular endothelial growth factor; *TGF*-*β* tumor growth factor β; *MMPs* matrix metalloproteinases

### Effect of anesthetic agents on immune function

#### Intravenous and volatile anesthetics

Intravenous anesthetics such as ketamine and thiopental produce multiple effects on immune system components. Unlike propofol, ketamine and thiopental suppress NK cell activity [34, 35]. Whereas ketamine induces human lymphocyte apoptosis via the mitochondrial pathway [36] and inhibits dendritic cell (DC) functional maturation [37], whereas thiopental protects against T-lymphocyte apoptosis through induction of heat shock proteins [38]. However, both of these intravenous anesthetics suppress the immune system in other ways: ketamine decreases production of pro-inflammatory cytokines such as IL-6 and tumor necrosis factor-α (TNF-α), and thiopental inhibits neutrophil function and suppresses activation of nuclear factor kappa B (NF-κB). This NF-κB suppression by thiopental is associated with inhibition of NF-κB-driven reporter gene activity, which includes T-lymphocyte activation as well as IL-2, IL-6, IL-8, and IFN-γ expression [39]. Thiopental also inhibits lipopolysaccharide-induced production of IL-1β, TNF-α, and IL-6 by monocytes [40]. Although intraperitoneal injection of midazolam impairs monocyte and neutrophil function, it does not affect cytotoxic T-lymphocyte (CTL) activity in a mouse model [41].

In contrast to other intravenous anesthetics, propofol increases CTL activity, decreases pro-inflammatory cytokines, and inhibits COX-2 and PGE_2_ functions [41–43]. Furthermore, propofol does not affect Th1/Th2, IL-2/IL-4, or CD4/CD8 T cell ratios, so surgery-induced immunosuppression is mitigated [44].

Volatile anesthetics also affect immune response. For example, halothane decreases NK cell activity and increases expression of hypoxia-inducible factor 1α (HIF-1α) [45, 46], and sevoflurane induces T-lymphocyte apoptosis and upregulates HIF-1α expression [46, 47]. Sevoflurane has also been shown to increase levels of pro-tumorigenic cytokines and MMPs in breast cancer surgery [48]. One study comparing desflurane to sevoflurane showed that sevoflurane decreases lymphocytes and NK cells while increasing leukocytes and neutrophils during abdominal surgery [49]. Similarly, isoflurane attenuates NK cell activity, induces T-lymphocyte and B-lymphocyte apoptosis, and decreases the Th1/Th2 ratio [44–46, 50]. Desflurane does not induce T-lymphocyte apoptosis [47].

#### Opioids and COX-2 inhibitors

Opioids usually inhibit T-lymphocyte proliferation [51]. Morphine suppresses NK cell activity and T cell differentiation, promotes lymphocyte apoptosis, and decreases toll-like receptor 4 (TLR4) expression on macrophages [51–54]. Likewise, fentanyl and sufentanil decrease NK cell activity but increase regulatory T cells [55, 56]. Sufentanil also inhibits leukocyte migration [57]. Alfentanil decreases NK cell activity [52], and remifentanil has demonstrated suppression of NK cell activity and lymphocyte proliferation in a rat model [58]. A comparison of sufentanil and remifentanil using target-controlled infusion during laparoscopic colorectal cancer resection showed that cortisol and IL-6 increased more in the remifentanil group and that the proportion of T cell subsets decreased more in the sufentanil group [59].

COX-2 induction, which is frequently observed in cancer, plays a role in immune evasion and resistance to the immune response. COX-2 inhibitors increase NK cytotoxicity and β-adrenergic antagonism while reducing postoperative LTR [31]. Additionally, combined β-adrenergic antagonism and COX-2 inhibition have been shown to eliminate LTR and decrease metastasis in animal models [60]. A selective COX-2 inhibitor can suppress PGE_2_ release and promote CTL immune responses that cause ovarian tumor regression [61]. Furthermore, a murine model has shown that celecoxib, a COX-2 inhibitor that reduces PGE_2_ levels, reduces and suppresses myeloid-derived suppressor cells (MDSCs); this in turn decreases reactive oxygen species and nitric oxide (NO) levels and reverses T cell tolerance [62]. Preoperative treatment with nonsteroidal anti-inflammatory drugs (NSAIDs) increases infiltration of activated immune cells into colorectal cancer tissue [63]. Of interest, a recent study showed that lidocaine at typical clinical concentrations enhanced NK cell activity against cancer cells in vitro via the release of lytic granules [64]. The overall effect of anesthetic agents on immune function is summarized in Table 2.

**Table 2:** Effect of anesthetic agent on immune function

Agent	Experimental data NK cell numbers (activity)	T-lymphocyte	Others	Clinical data
Intravenous				
Ketamine	Decrease [34, 35, 66]	Apoptosis [36]	Attenuation of proinflammatory cytokine (IL-6, TNF-α) production [35] Inhibition of functional maturation of DC [37] Suppression of neutrophil functions [35] Inhibition of NF-κB activation [39] Impairment of monocyte and neutrophil function [42] Decrease in secretion of proinflammatory cytokines [42] Inhibition of COX-2 and PGE_2_ 43	Inhibition of the lipopolysaccharide-induced production of IL-1β, TNF-α, and IL-6 by monocytes [40] No change in Th1/Th2 ratio [44]
Thiopental	Decrease [66]	Protection of apoptosis [38]		
Midazolam		No effect on CTL [41]		
Propofol	No suppression [66]	Increased activity on CTL [41]		
Volatile anesthetics				
Halothane	Decrease [45, 66]		Upregulation of HIF-1α [46] Upregulation of HIF-1α [46] B-lymphocyte apoptosis [50]	Increased levels of pro-tumorigenic cytokines and matrix metalloproteinases (MMPs) in breast cancer surgery [48] Decrease in Th1/Th2 ratio [44]
Sevoflurane	Decrease [49]	Apoptosis [47] /Decrease [49]		
Isoflurane	Attenuation [45]	Apoptosis [47]		
Nitrous oxide			Depression of neutrophil chemotaxis [18] Inhibition of formation of hematopoietic cells for tumor surveillance [52] Impairment of DNA, purine, and thymidylate synthesis [74]	No difference in cancer recurrence compared with oxygen [75]
Opioids				
Morphine	Suppression [52]	Suppressive effect on Th-cell differentiation [53] Increase in Tregs [56] Increase in Tregs [56] Decease in proliferation [58]	Inhibition of NF-κB binding [52] Decrease of TLR4 on MΦ [54] Promotion of apoptosis in lymphocytes and macrophages [77] Inhibitory effect on leucocyte migration [57]	Decrease in T-lymphocyte proliferation [51] Increase in IL-6; decrease in T cell subsets [59] Increase in IL-6; decrease in T cell subsets (less than sufentanil) [59]
Fentanyl	Decrease [34, 55]			
Sufentanil	Decrease [55]			
Alfentanil	Decrease [52]			
Remifentanil	Decrease [58]			
Others				
COX-2 inhibitor	Attenuation of NK cytotoxicity reduction using combined β-adrenergic antagonism [31]	Promotes CTL immune response [61] Reduced number of and suppressive function of MDSC [62]	Reduced postoperative LTR [31] Combination with β-adrenergic antagonist eliminates LTR [31] and decreases metastasis in animal models [60]	NSAIDs increase tumor infiltration by activated immune cells [63]
β-adrenergic antagonist				
Local anesthetics				
Lidocaine	Increase [64]			

*NK* natural killer; *IL*-*6* interleukin 6;*TNF*-*α* tumor necrosis factor-α; *DC* dendritic cell; *CTL* cytotoxic T-lymphocyte; *COX*-*2* cyclooxygenase 2; *PGE*_*2*_ prostaglandin E_2_; *HIF*-*1α* hypoxia inducible factor-1α; *MMPs* matrix metalloproteinases; *TLR4* toll-like receptor 4; *MΦ* macrophage; *NF*-*κB* nuclear factor kappa B; *LTR* lung tumor retention; *Tregs* CD4(+) CD25(+) Foxp3(+) regulatory T cells; *MDSC* myeloid-derived suppressor cells

### Effect of anesthetic agents on tumor development

#### Intravenous and volatile anesthetics

Treatment with intravenous anesthetics such as ketamine and thiopental stimulate lung and liver metastases in animal models [65], with one study showing that ketamine and thiopental increase LTR or lung metastasis via NK cell suppression in a rat model [66]. Similarly, the volatile anesthetic halothane can stimulate lung and liver metastases [65]. In contrast, sevoflurane suppresses hypoxia-inducible growth and metastasis of lung cancer cells by inhibiting HIF-1α, which is involved in the p38 mitogen-activated protein kinase (MAPK) signaling pathway [67]. Another study has shown that sevoflurane increases proliferation, migration, and invasion of estrogen receptor (ER)-positive breast cancer cells, as well as proliferation and migration of ER-negative cells [68]. Furthermore, serum from patients who received sevoflurane and an opioid for breast cancer surgery did not inhibit proliferation of ER-negative breast cancer cells, but serum from those receiving propofol and paravertebral anesthesia did inhibit proliferation [69].

Exposure to sevoflurane but not total intravenous anesthesia (TIVA) by propofol results in increased prosurvival proteins such as cytoplasmic HIF-2α and nuclear p38 MAPK in head and neck squamous cell carcinoma [70]. Isoflurane is associated with increased HIF-1α levels and increased prostate cancer cell proliferation and migration [71]. In contrast, isoflurane-induced HIF-1α activation is prevented by propofol, which is associated with partial reduction of malignant activities by cancer cells [71]. Additionally, tumor growth in inoculated in mice is suppressed by propofol, which may have immune-mediated antitumor effects [41]. Isoflurane increases the malignant potential of ovarian cancer cells through the upregulation of insulin-like growth factor (IGF)-1 and its receptor IGF-1R, as well as VEGF, angiopoietin-1, MMP-2, and MMP-9 [72]. Furthermore, isoflurane exposure leads to apoptotic resistance in human colon cancer cells through a caveolin-1-dependent mechanism [73]. Nitrous oxide (N_2_O) impairs DNA, purine, and thymidylate synthesis, which can itself cause of oncogenesis [74]. A tumor-bearing mouse model has shown that N_2_O suppresses chemotaxis, which may be the most potent stimulator of postsurgical lung and liver metastasis development [18, 65]. However, it is unlikely that N_2_O increases the risk of cancer recurrence compared to that of nitrogen after colorectal surgery [75].

#### Opioids and other agents

Commonly used opioid analgesics may affect tumor development through their modulation of cell proliferation and cell death [76–78]. It has been suggested that opioids suppress the immune response because various immune competent cells express opioid receptors and induce apoptosis during opioid alkaloid treatment. Tumor growth promotion is mediated through AKT and extracellular signal–regulated kinase (ERK) signaling cascades, whereas death-promoting effects are mediated through NF-κB inhibition, increased Fas expression, p53 stabilization, activation of p38, and c-Jun-N-terminal kinase (JNK) [79]. It is likely that opioid-induced cell proliferation and cell death depend on opioid concentration or exposure duration. Tumor growth promotion occurs with low concentrations or single doses of opioids, whereas growth inhibition occurs with chronic opioid use or relatively high drug concentrations [80].

Breast cancer cells treated with low morphine concentrations induce naloxone (NX)-sensitive, concentration-dependent increases in GTPase activity, with morphine signals being transmitted by opioid receptors via a G protein [81]. In contrast, the anti-proliferative effects of morphine are not eliminated by NX. Morphine-induced p53 phosphorylation and stabilization in breast cancer cells expressing wild type p53 causes increased production of p53-dependent proteins, including p21, Bax, and Fas [81]. These findings suggest that morphine may reduce growth of certain cancer cells through p53 activation. Additionally, morphine has been shown to inhibit expression and secretion of MMP-2 and MMP-9 in breast cancer cells in a time-dependent and concentration-dependent manner. This MMP activity is not reversible with NX, indicating that attenuation of MMP secretion by morphine is not mediated by opioid receptors, but is controlled by the NO system [82].

Based on preclinical and clinical studies, differences in recurrence rates for certain cancers may be due to immune suppression and direct effects of volatile anesthesia and opioids on cancer growth. Overexpression of the μ-opioid receptor (MOR), which promotes tumor growth and metastasis, is observed in several human cancers [83]. AKT and mTOR activation, cell proliferation, and extravasation are all related to MOR overexpression in a nude mouse model of non-small cell lung cancer (NSCLC) [84]. In addition, a potential direct effect of opiates has been observed in animal models that show MOR regulating tumorigenicity in Lewis lung carcinoma (LLC) [85]. Similarly, a study has shown the potential direct effect of opioids on MOR through growth factor-signaling proliferation, migration, and epithelial–mesenchymal transition during lung cancer progression [86]. Treatment with methylnaltrexone (MNTX), a peripheral opioid antagonist, inhibits LLC invasion and anchorage-independent growth, whereas continuous MNTX infusion decreases primary LLC tumor growth and lung metastasis [85]. Further, MNTX inhibits opioid-induced proliferation and migration of pulmonary microvascular endothelial cells through its effects on VEGF receptor phosphorylation and transactivation and inhibition of Rho A activation [87]. Clinically, MNTX treatment is associated with increased overall survival in patients with advanced cancer; this finding supports the hypothesis that MOR is involved in tumor progression and that MNTX may target MOR [88]. Because morphine reciprocally transactivates MOR and VEGF receptors, MOR-knockout mice do not grow significant lung cancer tumors; MNTX treatment markedly decreases tumor growth in experimental mouse models [89].

Morphine at clinical blood concentrations stimulates proliferation and angiogenesis of microvascular endothelial cells by activating MAPK/ERK phosphorylation using Gi/Go-coupled G protein receptors and NO. Effects include apoptotic inhibition of apoptosis through AKT activation and promotion of cell cycle progression through increased cyclin D1 [76]. Morphine at clinically useful doses promotes tumor neovascularization and progression in a xenograft model of a human breast tumor [76]. Similarly, clinical doses of morphine promote angiogenesis and tumor progression in ER-negative breast cancer cells in vitro and in vivo [90]. Morphine is also able to stimulate in vitro vascular endothelial cell proliferation, which is mediated by the MAPK pathway [91]. It is likely that MOR has an important role in angiogenesis and oncogenic signaling.

Preoperative and postoperative morphine administration for analgesia decreases the tumor promotion surgical effects in a rat model [92]. Preoperative and postoperative morphine treatment in rats significantly reduces surgery-induced corticosterone increases [93]. This finding suggests that preoperative morphine may play a key role in protecting against surgery-induced metastasis. Intraoperative opioid use has been associated with increased overall survival in patients with stage I but not stage II or III NSCLC [94].

Fentanyl has demonstrated antitumor-like effects in colorectal cancer cells in vitro. Its use is associated with decreased cell clone formation, and inhibition of cell migration and invasion through inhibition of negative regulation of E26 transformation–specific sequence-1 on serine/threonine kinase protein kinase B-raf (BRAF)-activated lncRNA [95]. Another study has shown that fentanyl inhibits tumor growth and cell invasion in colorectal cancer by downregulating miR-182 and MMP-9 expression using β-catenin [96]. A recent study showed that sufentanil does not affect the apoptosis rate or cell cycle distribution of colon and pancreatic cancer cells at clinical concentrations in vitro [97].

Although benefits of using RA to avoid opioids have been suggested by clinical trials, it is unclear whether benefits result from withholding opioids or adding RA. Morphine administration may be beneficial for pain control, but MOR is involved in tumor progression for certain cancer cell types. Opioids may play a crucial role in cancer metastasis and recurrence, but this effect varies by cancer cell type [98]. Prostaglandin E_2_, a soluble, tumor-derived angiogenic factor, is associated with VEGF-independent angiogenesis. PGE_2_ production in preclinical breast and colon cancer models is controlled by COX-2 expression, and COX-2 inhibition enhances VEGF blockade to inhibit angiogenesis, tumor growth, and metastasis to increase overall survival [99]. Previous case control studies show that selective COX-2 inhibitors reduce breast and colorectal cancer risk [100, 101], with the NSAID analgesic ketorolac being associated with a five-fold reduction in cancer relapse in the first few years after breast surgery [102]. Because transient and systemic inflammation following surgery may be involved in metastatic tumor seeding and angiogenesis, perioperative antiinflammatory agents may be used to block those effects.

#### Local anesthetics

Although local anesthetics suppress proliferation of several cancer cell types, their mechanism is unknown. Local anesthetics block voltage-gated sodium channels (VGSC), which are transmembrane proteins composed of one pore-forming α-unit and one or more auxiliary β-units. Cancer cells express an array of ion channels that their terminally differentiated counterparts do not [103]. VGSCs are highly expressed and active in breast, colon, and lung cancers, and local anesthetics that cause channel blockade may inhibit tumor growth. In fact, lidocaine, ropivacaine, and bupivacaine, which inhibit proliferation and differentiation, are cytotoxic to mesenchymal stem cells (MSCs) in vitro, and have key functions for tumor growth and metastatic formation in cancer cells [104].

Locally administered lidocaine directly inhibits epidermal growth factor receptor (EGFR), which is a potential target for anticancer drugs. Clinical concentrations of lidocaine have been shown to inhibit serum-induced and EGF-induced proliferation in human tongue cancer cells in association with tyrosine kinase activity of EGFR [105]. One study that assessed the direct effect of local anesthetics showed that clinically useful concentrations of lidocaine and bupivacaine induce apoptosis in breast cancer cells in vitro and in vivo, suggesting a potential benefit of local anesthetics for breast cancer surgery [106]. Lidocaine and tetracaine, which both inhibit kinesin motor proteins, reduce formation and function of tubulin micro-tentacles; thus, these drugs may have a novel ability to decrease metastatic spread in breast cancer cells [107]. Lidocaine use at clinical concentrations results in DNA demethylation from ER-positive and ER-negative breast cancer cells in vitro [108]. Although infiltrative anesthetics have the same membrane-stabilizing activity as lidocaine, they effectively inhibit the invasive ability of human cancer cells at the 5 mM to 20 mM concentrations used in surgery [109]. Lidocaine additionally blocks human cancer cell invasion through modulation of intracellular Ca^2+^ concentrations and inhibition of ectodomain shedding of heparin-binding epidermal growth factor from cell surfaces [109]. Furthermore, lidocaine, ropivacaine, and bupivacaine all reduce MSC proliferation at 100 μM concentrations by causing cell cycle delay or arrest at the G_0/1_-S phase; this feature is the reason why local anesthetics are used perioperatively for treatment of patients with cancer [96]. In contrast, ropivacaine and bupivacaine do cause apoptosis and cell cycle distribution at clinical concentrations for colon and pancreatic cancer cells in vitro; their only antitumor growth activity occurs at high concentrations [97]. Based on these findings, it is unlikely that the observed protective effects of RA on CMI result from direct effects on cancer cells. The overall effect of anesthetic agents on tumor development is summarized in Table 3.

**Table 3:** Effect of anesthetic agents on tumor development

Agent	Experimental data	Clinical data
Intravenous		
Ketamine	Stimulator of lung and liver metastasis [65] Increase in lung tumor retention or lung metastasis [66] Increase in lung tumor retention or lung metastasis [66] Inhibition of HIF-1α activation [71] Prevention of isoflurane-induced HIF-1α activation [71] Antitumor effect [18]	
Thiopental		
Propofol		
Volatile anesthetics		
Halothane	Stimulator of lung and liver metastasis [65] Suppression of hypoxia-induced growth and metastasis of lung cancer cells [35] Increased proliferation, migration, and invasion of breast cancer cells [77]	Serum from sevoflurane/opioid anesthesia-analgesia for breast cancer surgery attenuates the inhibition of breast cancer cell proliferation [69] Increased expression of pro-oncogenic protein markers in head and neck squamous cell carcinoma cells [70]
Sevoflurane		
Isoflurane	Upregulation of HIF-1α in prostate cancer cell line [71] Increase in malignant potential of ovarian cancer cells [72] Resistance against apoptosis via a Cav-1-dependent mechanism in cancer cells [73]	
Nitrous oxide	Suppression of neutrophil chemotaxis, potentially facilitating the spread of cancer [18] Potent stimulator of lung and liver metastasis [65]	No effect on colorectal carcinoma recurrence [87]
Opioids		
Morphine	Promotion of tumor growth (single-dose or low dose) [81] Involvement of MOR in tumor development [85–87] Promotion of tumor growth and metastasis by MOR overexpression [85] Proangiogenic and proliferative effects in breast cancer xenografts [76, 90] Increase in endothelial cell proliferation expressed with mu3 opioid receptor [91] Stimulation of Rho A and Src activation downstream of the VEGFR [88] Direct effect of morphine on breast cancer cell migration via *NET1* [68] Reduction in growth of certain tumors in part through activation of p53 [82] Attenuation of MMP secretion under the control of nitric oxide system [83] Beneficial effects on surgery-induced increases in metastasis by pre-surgical administration of morphine [93] Protective effect against metastasis development [34] Antitumor-like effects on colorectal cancer cells [95, 96] No change in apoptosis rate or cell cycle distribution at clinical concentrations [97]	Increase in MOR expression in patients with non-small cell lung cancer [86] and metastatic lung cancer [84] A possible adjuvant therapy of MNTX for patients with advanced cancer [88] Intraoperative opioid use is associated with decreased OS in stage I but not stage II-III NSCLC patients [94]
Fentanyl		
Sufentanil		
Others		
COX-2 inhibitor	Antitumor and antiangiogenic properties [99] Reduction of ketamine-induced lung metastasis [81]	Reduced risk of breast and colorectal cancer [100, 101] Use of COX-2 inhibitor was associated with one-fifth reduction in breast cancer recurrence [102]
β-adrenergic antagonist		
Local anesthetics		
Lidocaine	Antitumor effect of lidocaine via the inhibition of EGF/EGFR pathway in human tongue cancer cells [105] Apoptotic cell death by lidocaine and bupivacaine in breast cancer cells [106] Demethylation of DNA in breast cancer cell lines [108] Inhibition of cancer cell invasion [109] Reduced proliferation of mesenchymal stem cells [104] Decreased metastatic progression in breast tumor cells [107] Reduced proliferation of MSCs [104] No change in apoptosis rate or cell cycle distribution at clinical concentrations [97]	
Lidocaine/tetracaine		
Ropivacaine/bupivacaine		

*HIF*-*1α* hypoxia inducible factor-1α; *MOR* Mu-opioid receptor; *VEGFR* vascular endothelial growth factor receptor; *MNTX* methylnaltrexone; *MMP* matrix metalloproteinase; *NSCLC* non-small cell lung cancer; *COX*-*2* cyclooxygenase-2; *EGF* epidermal growth factor; *EGFR* epidermal growth factor receptor; *MSCs* mesenchymal stem cells

### Potential for cancer recurrence caused by surgery and anesthetic-induced immunosuppression

In general, cancer is considered as a systemic disease with circulating tumor cells and micro-metastases present at initial diagnosis. Surgery and anesthetic-induced immunosuppression activate HPA-axis and SNS responses, which in turn increase neuroendocrine mediators. These mediators promote metastasis to regional lymph nodes and distant sites from residual or circulating tumor cells, and stimulate growth of preexisting, dormant micro-metastases through immunosuppression (Fig. 2). During this process, cancer cells must escape immunoediting by NK cells and CTLs to establish themselves at distant sites and proceed to angiogenesis.

**Fig. 2:** Hypothesis to explain cancer metastasis and recurrence caused by surgery- and anesthetic-induced immunosuppression in the perioperative period. Surgery, anesthesia, and analgesia stimulate the HPA-axis and SNS during the perioperative period. Activated neuroendocrine mediators lead to increases in several immunosuppressive soluble factors that promote tumor progression and metastasis, resulting in increase of cancer recurrence. Combined regional anesthesia with propofol decreases anesthesia-induced immunosuppression and avoids volatile anesthetics and opioids, which may increase the risk of cancer recurrence

Tumor dormancy, often described as “cancer without disease,” is the poorly understood phenomenon by which quiescent cancer cells exist but do not produce clinical disease [110]. Distant recurrence appearing months or years after surgical resection have been described as dormant metastases, which are clinically undetectable, pre-existing disease foci that then become clinically detectable. Two potential explanations for tumor dormancy are 1) lack of angiogenic activity; and 2) immunologic equilibrium between tumor and host immunity, which prevents further tumor growth in the microenvironment. Because neuroendocrine mediators regulate tumor progression biology and act as endogenous angiogenesis modulators of reactivation from dormancy, HPA-axis and SNS neuroendocrine dynamics may be responsible for loss of tumor dormancy [6]. Thus, surgery-induced and anesthetic-induced immunosuppression may promote cancer recurrence through HPA-axis and SNS activation during the perioperative period in patients with cancer.

## Conclusion

Currently available preclinical studies suggest that anesthetic-induced immunosuppression may promote cancer recurrence in patients with certain types of cancer. Volatile anesthetic agents and morphine or synthetic opioids produce diverse effects on cancer cells that depend on dose, duration, and timing of use. Nevertheless, locoregional anesthesia and propofol-based anesthesia seem to reduce surgical stress, perioperative immunosuppression, and angiogenesis compared to general anesthesia with volatile anesthetics and opioids. Although a causal link between anesthetics, immune function, survival, and residual disease remains to be elucidated, several ongoing prospective RCTs should provide more definitive information about the effects of anesthesia on cancer recurrence after surgery.

## Abbreviations

NK: natural killer
HPA: hypothalamic–pituitary–adrenal
SNS: sympathetic nervous system
CMI: cell-mediated immunity
PGE_2_: prostaglandin E_2_
IL: interleukin
TGF-β: transforming growth factor beta
VEGF: vascular endothelial growth factor
RA: regional anesthesia
RCT: srandomized controlled trials
MMP: matrix metalloproteinase
LTR: lung tumor retention
COX: cyclooxygenase
PD-1: programmed death-1
PD-L1: programmed death–ligand 1
IFN-γ: interferon-γ
NF-κB: nuclear factor kappa B
CTL: cytotoxic T-lymphocyte
HIF-1α: hypoxia-inducible factor 1α
MDSCs: myeloid-derived suppressor cells
NO: nitric oxide
NSAIDs: nonsteroidal anti-inflammatory drugs
MAPK: mitogen-activated protein kinase
ER: estrogen receptor
TIVA: total intravenous anesthesia
IGF: insulin-like growth factor
ERK: extracellular signal–regulated kinase
N_2_O: nitrous oxide
NX: naloxone
MOR: μ-opioid receptor
NSCLC: non-small cell lung cancer
LLC: Lewis lung carcinoma
MNTX: methylnaltrexone
VGSC: voltage-gated sodium channels
MSCs: mesenchymal stem cells
EGFR: epidermal growth factor receptors

## References

[1] Lloyd JM, McIver CM, Stephenson SA, Hewett PJ, Rieger N, Hardingham JE (2006). Identification of early-stage colorectal cancer patients at risk of relapse post-resection by immunobead reverse transcription-PCR analysis of peritoneal lavage fluid for malignant cells. Clin Cancer Res.

[2] Looney M, Doran P, Buggy DJ (2010). Effect of anesthetic technique on serum vascular endothelial growth factor C and transforming growth factor β in women undergoing anesthesia and surgery for breast cancer. Anesthesiology.

[3] Thaker PH, Han LY, Kamat AA, Arevalo JM, Takahashi R, Lu C (2006). Chronic stress promotes tumor growth and angiogenesis in a mouse model of ovarian carcinoma. Nat Med.

[4] Baum M, Demicheli R, Hrushesky W, Retsky M (2005). Does surgery unfavourably perturb the “natural history” of early breast cancer by accelerating the appearance of distant metastases?. Eur J Cancer.

[5] Retsky M, Demicheli R, Hrushesky WJ (2005). Does surgery induce angiogenesis in breast cancer? Indirect evidence from relapse pattern and mammography paradox. Int J Surg..

[6] Zappalà G, McDonald PG, Cole SW (2013). Tumor dormancy and the neuroendocrine system: an undisclosed connection?. Cancer Metastasis Rev.

[7] Sood AK, Bhatty R, Kamat AA, Landen CN, Han L, Thaker PH (2006). Stress hormone-mediated invasion of ovarian cancer cells. Clin Cancer Res.

[8] Wong HP, Ho JW, Koo MW, Yu L, Wu WK, Lam EK (2011). Effects of adrenaline in human colon adenocarcinoma HT-29 cells. Life Sci.

[9] Bernabé DG, Tamae AC, Biasoli ÉR, Oliveira SH (2011). Stress hormones increase cell proliferation and regulates interleukin-6 secretion in human oral squamous cell carcinoma cells. Brain Behav Immun.

[10] Yang EV, Kim SJ, Donovan EL, Chen M, Gross AC, Webster Marketon JI (2009). Norepinephrine upregulates VEGF, IL-8, and IL-6 expression in human melanoma tumor cell lines: implications for stress-related enhancement of tumor progression. Brain Behav Immun.

[11] Calcagni E, Elenkov I (2006). Stress system activity, innate and T helper cytokines, and susceptibility to immune-related diseases. Ann N.Y Acad Sci.

[12] Gottschalk A, Sharma S, Ford J, Durieux ME, Tiouririne M (2010). Review article: the role of the perioperative period in recurrence after cancer surgery. Anesth Analg.

[13] Neeman E, Ben-Eliyahu S (2013). Surgery and stress promote cancer metastasis: new outlooks on perioperative mediating mechanisms and immune involvement. Brain Behav Immun.

[14] Horowitz M, Neeman E, Sharon E, Ben-Eliyahu S (2015). Exploiting the critical perioperative period to improve long-term cancer outcomes. Nat Rev Clin Oncol..

[15] Kim R (2017). Anesthetic technique and cancer recurrence in oncologic. surgery: unraveling the puzzle. Cancer Metastasis Rev.

[16] Kim R, Emi M, Tanabe K, Arihiro K (2006). Tumor-driven evolution of immunosuppressive networks during malignant progression. Cancer Res.

[17] Kavanagh T, Buggy DJ (2012). Can anaesthetic technique effect postoperative outcome?. Curr Opin Anaesthesiol..

[18] Kurosawa S, Kato M (2008). Anesthetics, immune cells, and immune responses. J Anesth..

[19] Lee BM, Cata JP (2015). Impact of anesthesia on cancer recurrence. Rev Esp Anestesiol Reanim.

[20] Coffey JC, Wang JH, Smith MJ, Bouchier-Hayes D, Cotter TG, Redmond HP (2003). Excisional surgery for cancer cure: therapy at a cost. Lancet Oncol..

[21] Yamaguchi K, Takagi Y, Aoki S, Futamura M, Saji S (2000). Significant detection of circulating cancer cells in the blood by reverse transcriptase-polymerase chain reaction during colorectal cancer resection. Ann Surg.

[22] Mao L, Lin S, Lin J (2013). The effects of anesthetics on tumor progression. Int J Physiol Pathophysiol Pharmacol..

[23] Zhao T, Xia WH, Zheng MQ, Lu CQ, Han X, Sun YJ (2008). Surgical excision promotes tumor growth and metastasis by promoting expression of MMP-9 and VEGF in a breast cancer model. Exp Oncol..

[24] Wang HL, Ning T, Li M, Lu ZJ, Yan X, Peng Q (2011). Effect of endostatin on preventing postoperative progression of distant metastasis in a murine lung cancer model. Tumori.

[25] Demicheli R, Miceli R, Moliterni A, Zambetti M, Hrushesky WJ, Retsky MW (2005). Breast cancer recurrence dynamics following adjuvant CMF is consistent with tumor dormancy and mastectomy-driven acceleration of the metastatic process. Ann Oncol.

[26] Wu FP, Westphal JR, Hoekman K, Mels AK, Statius Muller MG, de Waal RW (2004). The effects of surgery, with or without rhGM-CSF, on the angiogenic profile of patients treated for colorectal carcinoma. Cytokine.

[27] Peeters CF, de Geus LF, Westphal JR, de Waal RM, Ruiter DJ, Wobbes T (2005). Decrease in circulating anti-angiogenic factors (angiostatin and endostatin) after surgical removal of primary colorectal carcinoma coincides with increased metabolic activity of liver metastases. Surgery.

[28] Oliver RT (1995). Does surgery disseminate or accelerate cancer?. Lancet.

[29] Ben-Eliyahu S, Page GG, Yirmiya R, Shakhar G (1999). Evidence that stress and surgical interventions promote tumor development by suppressing natural killer cell activity. Int J Cancer.

[30] Heaney A, Buggy DJ (2012). Can anaesthetic and analgesic techniques affect cancer recurrence or metastasis?. Br J Anaesth.

[31] Benish M, Bartal I, Goldfarb Y, Levi B, Avraham R, Raz A (2008). Perioperative use of beta-blockers and COX-2 inhibitors may improve immune competence and reduce the risk of tumor metastasis. Ann Surg Oncol.

[32] Xu P, Zhang P, Sun Z, Wang Y, Chen J, Miao C (2015). Surgical trauma induces postoperative T-cell dysfunction in lung cancer patients through the programmed death-1 pathway. Cancer Immunol Immunother.

[33] Lin E, Calvano SE, Lowry SF (2000). Inflammatory cytokines and cell response in surgery. Surgery.

[34] Forget P, Collet V, Lavand’homme P, De Kock M (2010). Does analgesia and condition influence immunity after surgery? Effects of fentanyl, ketamine and clonidine on natural killer activity at different ages. Eur J Anaesthesiol.

[35] Nishina K, Akamatsu H, Mikawa K, Shiga M, Maekawa N, Obara H (1998). The inhibitory effects of thiopental, midazolam, and ketamine on human neutrophil functions. Anesth Analg.

[36] Braun S, Gaza N, Werdehausen R, Hermanns H, Bauer I, Durieux ME (2010). Ketamine induces apoptosis via the mitochondrial pathway in human lymphocytes and neuronal cells. Br J Anaesth.

[37] Ohta N, Ohashi Y, Fujino Y (2009). Ketamine inhibits maturation of bone marrow-derived dendritic cells and priming of the Th1-type immune response. Anesth Analg.

[38] Roesslein M, Schibilsky D, Muller L, Goebel U, Schwer C, Humar M (2008). Thiopental protects human T lymphocytes from apoptosis in vitro via the expression of heat shock protein 70. J Pharmacol Exp Ther.

[39] Loop T, Liu Z, Humar M, Hoetzel A, Benzing A, Pahl HL (2002). Thiopental inhibits the activation of nuclear factor kappa B. Anesthesiology.

[40] Taupin V, Jayais P, Descamps-Latscha B, Cazalaa JB, Barrier G, Bach JF (1991). Benzodiazepine anesthesia in humans modulates the interleukin-1 beta, tumor necrosis factor-alpha and interleukin-6 responses of blood monocytes. J Neuroimmunol.

[41] Kushida A, Inada T, Shingu K (2007). Enhancement of antitumor immunity after propofol treatment in mice. Immunopharmacol Immunotoxicol.

[42] Vanlersberghe C, Camu F (2008). Propofol. Handb Exp Pharmacol.

[43] Inada T, Kubo K, Shingu K (2011). Possible link between cyclooxygenase-inhibiting and antitumor properties of propofol. J Anesth..

[44] Inada T, Yamanouchi Y, Jomura S, Sakamoto S, Takahashi M, Kambara T (2004). Effect of propofol and isoflurane anaesthesia on the immune response to surgery. Anaesthesia.

[45] Markovic SN, Knight PR, Murasko DM (1993). Inhibition of interferon stimulation of natural killer cell activity in mice anesthetized with halothane or isoflurane. Anesthesiology.

[46] Tavare AN, Perry NJ, Benzonana LL, Takata M, Ma D (2012). Cancer recurrence after surgery: direct and indirect effects of anesthetic agents. Int J Cancer.

[47] Loop T, Dovi-Akue D, Frick M, Roesslein M, Egger L, Humar M (2005). Volatile anesthetics induce caspase-dependent, mitochondria-mediated apoptosis in human T lymphocytes in vitro. Anesthesiology.

[48] Deegan CA, Murray D, Doran P, Moriarty DC, Sessler DI, Mascha E (2010). Anesthetic technique and the cytokine and matrix metalloproteinase response to primary breast cancer surgery. Reg Anesth Pain Med.

[49] Pirbudak Cocelli L, Ugur MG, Karadasli H (2012). Comparison of effects of low-flow sevoflurane and desflurane anesthesia on neutrophil and T-cell populations. Curr Ther Res Clin Exp..

[50] Wei H, Liang G, Yang H, Wang Q, Hawkins B, Madesh M (2008). The common inhalational anesthetic isoflurane induces apoptosis via activation of inositol 1,4,5-trisphosphate receptors. Anesthesiology.

[51] Sacerdote P, Bianchi M, Gaspani L, Manfredi B, Maucione A, Terno G (2000). The effects of tramadol and morphine on immune responses and pain after surgery in cancer patients. Anesth Analg.

[52] Das J, Kumar S, Khanna S, Mehta Y (2014). Are we causing the recurrence-impact of perioperative period on long-term cancer prognosis: review of current evidence and practice. J Anaesthesiol Clin Pharmacol..

[53] Gao M, Sun J, Jin W, Qian Y (2012). Morphine, but not ketamine, decreases the ratio of Th1/Th2 in CD4-positive cells through T-bet and GATA3. Inflammation.

[54] Franchi S, Moretti S, Castelli M, Lattuada D, Scavullo C, Panerai AE (2012). Mu opioid receptor activation modulates Toll like receptor 4 in murine macrophages. Brain Behav Immun.

[55] Shavit Y, Ben-Eliyahu S, Zeidel A, Beilin B (2004). Effects of fentanyl on natural killer cell activity and on resistance to tumor metastasis in rats. Dose and timing study. Neuroimmunomodulation.

[56] Gong L, Qin Q, Zhou L, Ouyang W, Li Y, Wu Y (2014). Effects of fentanyl anesthesia and sufentanil anesthesia on regulatory T cells frequencies. Int J Clin Exp Pathol..

[57] Hofbauer R, Moser D, Salfinger H, Frass M, Kapiotis S (1998). Sufentanil inhibits migration of human leukocytes through human endothelial cell monolayers. Anesth Analg.

[58] Sacerdote P, Gaspani L, Rossoni G, Panerai AE, Bianchi M (2001). Effect of the opioid remifentanil on cellular immune response in the rat. Int Immunopharmacol.

[59] Qi Y, Yao X, Zhang B, Du X (2016). Comparison of recovery effect for sufentanil and remifentanil anesthesia with TCI in laparoscopic radical resection during colorectal cancer. Oncol Lett..

[60] Glasner A, Avraham R, Rosenne E, Benish M, Zmora O, Shemer S (2010). Improving survival rates in two models of spontaneous postoperative metastasis in mice by combined administration of a beta-adrenergic antagonist and a cyclooxygenase-2 inhibitor. J Immunol..

[61] Wang X, Liang Y, Wang J, Wang M (2013). Effect of NS-398, a cyclooxygenase-2 selective inhibitor, on the cytotoxicity of cytotoxic T lymphocytes to ovarian carcinoma cells. Tumour Biol.

[62] Veltman JD, Lambers ME, van Nimwegen M, Hendriks RW, Hoogsteden HC, Aerts JG (2010). COX-2 inhibition improves immunotherapy and is associated with decreased numbers of myeloid-derived suppressor cells in mesothelioma. Celecoxib influences MDSC function. BMC Cancer.

[63] Lönnroth C, Andersson M, Arvidsson A, Nordgren S, Brevinge H, Lagerstedt K (2008). Preoperative treatment with a non-steroidal anti-inflammatory drug (NSAID) increases tumor tissue infiltration of seemingly activated immune cells in colorectal cancer. Cancer Immun..

[64] Ramirez MF, Tran P, Cata JP (2015). The effect of clinically therapeutic plasma concentrations of lidocaine on natural killer cell cytotoxicity. Reg Anesth Pain Med.

[65] Shapiro J, Jersky J, Katzav S, Feldman M, Segal S (1981). Anesthetic drugs accelerate the progression of postoperative metastases of mouse tumors. J Clin Invest..

[66] Melamed R, Bar-Yosef S, Shakhar G, Shakhar K, Ben-Eliyahu S (2003). Suppression of natural killer cell activity and promotion of tumor metastasis by ketamine, thiopental, and halothane, but not by propofol: mediating mechanisms and prophylactic measures. Anesth Analg.

[67] Liang H, Yang CX, Zhang B, Wang HB, Liu HZ, Lai XH (2015). Sevoflurane suppresses hypoxia-induced growth and metastasis of lung cancer cells via inhibiting hypoxia-inducible factor-1α. J Anesth..

[68] Ecimovic P, McHugh B, Murray D, Doran P, Buggy DJ (2013). Effects of sevoflurane on breast cancer cell function in vitro. Anticancer Res.

[69] Deegan CA, Murray D, Doran P, Ecimovic P, Moriarty DC, Buggy DJ (2009). Effect of anaesthetic technique on oestrogen receptor-negative breast cancer cell function in vitro. Br J Anaesth.

[70] Ferrell JK, Cattano D, Brown RE, Patel CB, Karni RJ (2015). The effects of anesthesia on the morphoproteomic expression of head and neck squamous cell carcinoma: a pilot study. Transl Res..

[71] Huang H, Benzonana LL, Zhao H, Watts HR, Perry NJ, Bevan C (2014). Prostate cancer cell malignancy via modulation of HIF-1α pathway with isoflurane and propofol alone and in combination. Br J Cancer.

[72] Luo X, Zhao H, Hennah L, Ning J, Liu J, Tu H (2015). Impact of isoflurane on malignant capability of ovarian cancer in vitro. Br J Anaesth.

[73] Kawaraguchi Y, Horikawa YT, Murphy AN, Murray F, Miyanohara A, Ali SS (2011). Volatile anesthetics protect cancer cells against tumor necrosis factor-related apoptosis-inducing ligand-induced apoptosis via caveolins. Anesthesiology.

[74] Moudgil GC, Gordon J, Forrest JB (1984). Comparative effects of volatile anaesthetic agents and nitrous oxide on human leucocyte chemotaxis in vitro. Can Anaesth Soc J..

[75] Fleischmann E, Marschalek C, Schlemitz K, Dalton JE, Gruenberger T, Herbst F (2009). Nitrous oxide may not increase the risk of cancer recurrence after colorectal surgery: a follow-up of a randomized controlled trial. BMC Anesthesiol..

[76] Gupta K, Kshirsagar S, Chang L, Schwartz R, Law PY, Yee D (2002). Morphine stimulates angiogenesis by activating proangiogenic and survival-promoting signaling and promotes breast tumor growth. Cancer Res.

[77] Singhal PC, Sharma P, Kapasi AA, Reddy K, Franki N, Gibbons N (1998). Morphine enhances macrophage apoptosis. J Immunol..

[78] Hatzoglou A, Bakogeorgou E, Castanas E (1996). The antiproliferative effect of opioid receptor agonists on the T47D human breast cancer cell line, is partially mediated through opioid receptors. Eur J Pharmacol.

[79] Tegeder I, Geisslinger G (2004). Opioids as modulators of cell death and survival–unraveling mechanisms and revealing new indications. Pharmacol Rev.

[80] Lin X, Wang YJ, Li Q, Hou YY, Hong MH, Cao YL (2009). Chronic high-dose morphine treatment promotes SH-SY5Y cell apoptosis via c-Jun N-terminal kinase-mediated activation of mitochondria-dependent pathway. FEBS J.

[81] Tegeder I, Grösch S, Schmidtko A, Häussler A, Schmidt H, Niederberger E (2003). G protein-independent G1 cell cycle block and apoptosis with morphine in adenocarcinoma cells: involvement of p53 phosphorylation. Cancer Res.

[82] Gach K, Szemraj J, Wyrębska A, Janecka A (2011). The influence of opioids on matrix metalloproteinase-2 and -9 secretion and mRNA levels in MCF-7 breast cancer cell line. Mol Biol Rep.

[83] Singleton PA, Mirzapoiazova T, Hasina R, Salgia R, Moss J (2014). Increased μ-opioid receptor expression in metastatic lung cancer. Br J Anaesth.

[84] Lennon FE, Mirzapoiazova T, Mambetsariev B, Salgia R, Moss J, Singleton PA (2012). Overexpression of the μ-opioid receptor in human non-small cell lung cancer promotes Akt and mTOR activation, tumor growth, and metastasis. Anesthesiology.

[85] Mathew B, Lennon FE, Siegler J, Mirzapoiazova T, Mambetsariev N, Sammani S (2011). The novel role of the mu opioid receptor in lung cancer progression: a laboratory investigation. Anesth Analg.

[86] Lennon FE, Mirzapoiazova T, Mambetsariev B, Poroyko VA, Salgia R, Moss J (2014). The Mu opioid receptor promotes opioid and growth factor-induced proliferation, migration and Epithelial Mesenchymal Transition (EMT) in human lung cancer. PLoS ONE.

[87] Singleton PA, Lingen MW, Fekete MJ, Garcia JG, Moss J (2006). Methylnaltrexone inhibits opiate and VEGF-induced angiogenesis: role of receptor transactivation. Microvasc Res.

[88] Janku F, Johnson LK, Karp DD, Atkins JT, Singleton PA, Moss J (2016). Treatment with methylnaltrexone is associated with increased survival in patients with advanced cancer. Ann Oncol.

[89] Singleton PA, Moss J (2010). Effect of perioperative opioids on cancer recurrence: a hypothesis. Future Oncol..

[90] Bimonte S, Barbieri A, Rea D, Palma G, Luciano A, Cuomo A (2015). Morphine promotes tumor angiogenesis and increases breast cancer progression. Biomed Res Int..

[91] Leo S, Nuydens R, Meert TF (2009). Opioid-induced proliferation of vascular endothelial cells. J Pain Res..

[92] Page GG, Ben-Eliyahu S, Yirmiya R, Liebeskind JC (1993). Morphine attenuates surgery-induced enhancement of metastatic colonization in rats. Pain.

[93] Page GG, McDonald JS, Ben-Eliyahu S (1998). Pre-operative versus postoperative administration of morphine: impact on the neuroendocrine, behavioural, and metastatic-enhancing effects of surgery. Br J Anaesth.

[94] Cata JP, Keerty V, Keerty D, Feng L, Norman PH, Gottumukkala V (2014). A retrospective analysis of the effect of intraoperative opioid dose on cancer recurrence after non-small cell lung cancer resection. Cancer Med.

[95] Li AX, Xin WQ, Ma CG (2015). Fentanyl inhibits the invasion and migration of colorectal cancer cells via inhibiting the negative regulation of Ets-1 on BANCR. Biochem Biophys Res Commun.

[96] Zhang XL, Chen ML, Zhou SL (2015). Fentanyl inhibits proliferation and invasion of colorectal cancer via β-catenin. Int J Clin Exp Pathol..

[97] Bundscherer A, Malsy M, Gebhardt K, Metterlein T, Plank C, Wiese CH (2015). Effects of ropivacaine, bupivacaine and sufentanil in colon and pancreatic cancer cells in vitro. Pharmacol Res.

[98] Juneja R (2014). Opioids and cancer recurrence. Curr Opin Support Palliat Care.

[99] Xu L, Stevens J, Hilton MB, Seaman S, Conrads TP, Veenstra TD (2014). COX-2 inhibition potentiates antiangiogenic cancer therapy and prevents metastasis in preclinical models. Sci Transl Med..

[100] Harris RE, Beebe-Donk J, Alshafie GA (2006). Reduction in the risk of human breast cancer by selective cyclooxygenase-2 (COX-2) inhibitors. BMC Cancer.

[101] Yang YH, Yang YH, Cheng CL, Ho PS, Ko YC (2012). The role of chemoprevention by selective cyclooxygenase-2 inhibitors in colorectal cancer patients—a population-based study. BMC Cancer.

[102] Retsky M, Rogers R, Demicheli R, Hrushesky WJ, Gukas I, Vaidya JS (2012). NSAID analgesic ketorolac used perioperatively may suppress early breast cancer relapse: particular relevance to triple negative subgroup. Breast Cancer Res Treat.

[103] Li M, Xiong ZG (2011). Ion channels as targets for cancer therapy. Int J Physiol Pathophysiol Pharmacol..

[104] Lucchinetti E, Awad AE, Rahman M, Feng J, Lou PH, Zhang L (2012). Antiproliferative effects of local anesthetics on mesenchymal stem cells: potential implications for tumor spreading and wound healing. Anesthesiology.

[105] Sakaguchi M, Kuroda Y, Hirose M (2006). The antiproliferative effect of lidocaine on human tongue cancer cells with inhibition of the activity of epidermal growth factor receptor. Anesth Analg.

[106] Chang YC, Liu CL, Chen MJ, Hsu YW, Chen SN, Lin CH (2014). Local anesthetics induce apoptosis in human breast tumor cells. Anesth Analg.

[107] Yoon JR, Whipple RA, Balzer EM, Cho EH, Matrone MA, Peckham M (2011). Local anesthetics inhibit kinesin motility and microtentacle protrusions in human epithelial and breast tumor cells. Breast Cancer Res Treat.

[108] Lirk P, Berger R, Hollmann MW, Fiegl H (2012). Lidocaine time- and dose-dependently demethylates deoxyribonucleic acid in breast cancer cell lines in vitro. Br J Anaesth.

[109] Mammoto T, Higashiyama S, Mukai M, Mammoto A, Ayaki M, Mashimo T (2002). Infiltration anesthetic lidocaine inhibits cancer cell invasion by modulating ectodomain shedding of heparin-binding epidermal growth factor-like growth factor (HB-EGF). J Cell Physiol.

[110] John A, Tuszynski G (2001). The role of matrix metalloproteinases in tumor angiogenesis and tumor metastasis. Pathol Oncol Res..

